The article "Effect Analysis of Lung Rehabilitation Training in 5A Nursing Mode for Elderly Patients with COPD Based on X-Ray" was published in 2022. Journal: Comput Math Methods Med.

# Effect Analysis of Lung Rehabilitation Training in 5A Nursing Mode for Elderly Patients with COPD Based on X-Ray

**DOI:** 10.1155/2022/1963426

**Published:** 2022-06-13

**Authors:** Peihong Xu, Wei Zheng, Yanjun Zhu

**Affiliations:** Department of Respiratory, The Affiliated People's Hospital of Ningbo University, Ningbo, 315040 Zhejiang, China

## Abstract

This study was aimed at evaluating the application effect of pulmonary rehabilitation training under 5A nursing mode based on X-ray in elderly patients with chronic obstructive pulmonary disease (COPD). Then, 84 elderly patients with chronic obstructive emphysema were selected as the research subjects. COPD knowledge level questionnaire, caregiver self-efficacy scale (CSES), COPD assessment test (CAT), and 6-minute walking experiment (6MWD) were adopted, and the clinical application effect of pulmonary rehabilitation training and conventional nursing under 5A nursing mode was comprehensively compared. The results show that after two and four months of intervention, the average score of COPD knowledge level questionnaire in the test group was 27.43 points and 30.08 points, respectively, higher than that in the control group (*P* < 0.05). After two and four months of intervention, the number of patients with good compliance in the test group was remarkably improved, and the severity of airflow restriction in the test group was slower than that in the control group. In short, pulmonary rehabilitation training under 5A nursing mode based on X-ray can effectively improve the disease knowledge level, self-efficacy, and pulmonary rehabilitation training compliance of elderly COPD patients, which played an important role in improving the quality of life of patients and alleviating the degree of dyspnea of patients.

## 1. Introduction

Chronic obstructive pulmonary disease (COPD) is a common respiratory disorder. The disease has a high incidence in the elderly population and has a high risk of disability and death, causing serious economic burden to the families of patients, which has become a public health problem of major concern in China [1–3]. Studies pointed out that the global incidence of COPD in recent years is 4%~10%, and the incidence of COPD in China's population over 40 years old is about 8.2%. The incidence rate of the elderly group over 60 years old is about 27%, and the mortality rate is as high as 17.6% [4, 5]. Therefore, it is of great significance to improve the clinical diagnosis and treatment level of COPD, put forward reasonable prevention programs, and reduce the economic burden of patients' families [6, 7].

5A nursing model is a new nursing model proposed by the International Cancer Society, including assessment, consensus, assistance, advice, and follow-up [8–11]. 5A nursing mode is often used for management of diabetes and chronic anemia. Puschel et al. (2008) implemented a smoking cessation management program based on 5A nursing mode for female smokers. The results showed that the amount of smoking of the target population decreased with the extension of intervention time [12–15]. Although 5A nursing mode has been widely applied in cancer management and diabetes management in China, it is seldom applied in pulmonary rehabilitation training for elderly COPD patients.

At present, the commonly used imaging examination methods for COPD include chest X-ray plain film, computed tomography (CT), and pulmonary function examination. Pulmonary function examination is the main method to evaluate the severity of COPD, but it has great limitations. On the one hand, this method requires patients to have a high ability to cooperate, while elderly patients have poor ability to cooperate and even cannot tolerate it in severe cases. On the other hand, pulmonary function examination can only evaluate the overall lung condition of patients, and cannot effectively reflect the specific clinical symptoms of patients [16–19].

In summary, COPD has a high incidence and mortality rate in the elderly population. How to improve the clinical diagnosis and treatment level of COPD is of great clinical significance. 5A nursing mode is rarely used in pulmonary rehabilitation training of COPD patients. In this study, a total of 84 patients with chronic obstructive emphysema were randomly divided into an experimental group (pulmonary rehabilitation nursing under 5A mode) and a control group (routine nursing), 42 cases in each group. The effects of 5A-mode-based lung rehabilitation training on elderly patients with COPD were comprehensively evaluated through questionnaire on the knowledge level of chronic obstructive pulmonary disease, caregiver self-efficacy scale (CSES), chronic obstructive pulmonary disease assessment test (CAT), 6-minute walk test (6MWD), and X-ray image scanning.

## 2. Materials and Methods

### 2.1. Research Objects and Grouping

A total of 84 patients with chronic obstructive emphysema admitted to hospital from June 2020 to June 2021 were selected as the research objects, and the patients were randomly divided into test group and control group, with 42 patients in each group. Patients in the test group and control group were 60-80 years old. There were no substantial differences in gender, age, and education level between the two groups (*P* < 0.05). Inclusion criteria: (i) patients aged ≥60 years; (ii) patients conformed to the *Guidelines for Diagnosis and Treatment of Chronic Obstructive Pulmonary Diseases* [20]; (iii) patient's pulmonary function was grades II to III; and (iv) patients had good compliance and could cooperate with the study. Exclusion criteria: (i) patients cannot complete pulmonary rehabilitation training due to their own diseases; (ii) patients with malignant tumor or serious blood diseases; and (iii) patients with a history of cognitive impairment or mental illness. This study had been approved by the ethics committee of the hospital.

### 2.2. Intervention Measures

The control group received routine nursing, including oxygen therapy, medication guidance, health education, smoking cessation guidance, and diet guidance.

Based on the routine treatment of patients in the test group, a pulmonary rehabilitation group was established. The team was composed of respiratory physicians, nurses, and nutritionists.

In the assessment phase, the pulmonary rehabilitation team comprehensively evaluated the patient's specific condition within two days of admission. General clinical data, COPD severity, disease-related knowledge, family economic status, self-efficacy, compliance, and exercise tolerance were collected. Through the collected information, the rehabilitation team negotiated and formulated training programs according to the patient's own situation. The main assessment scales used were knowledge level questionnaire, self-efficacy scale (CSES), and COPD assessment questionnaire (CAT) (Table 1).

Recommendation stage: health education was conducted for patients and their families two days before admission, one week after hospitalization, and two days before discharge.

Consensus stage: medical staff set up a rehabilitation goal for patients and encouraged patients and their families to actively carry out pulmonary rehabilitation training by using successful cases in the process of pulmonary rehabilitation training.

Assistance stage: the Richmond Agitation-Sedation Scale (RASS) and MAC muscle strength assessment scale were adopted, combined with recommended guidelines, for pulmonary rehabilitation training, as shown in Table 2.

During the follow-up period, the pulmonary rehabilitation team established a COPD service platform using the Internet to answer questions for patients after discharge. The patient was followed up by telephone within two days after discharge. One follow-up visit was paid per month within two months after discharge. Follow-up visits were performed every two months after discharge. Each follow-up lasted 25-35 minutes.

### 2.3. Imaging Examination and Image Reconstruction

The patient was placed in the supine position, arms were raised, the positioning film was scanned first, and then, the scanning range (from the lung apex to the lung base) was determined on the positioning film. It should scan while holding your breath after taking a deep breath or holding your breath after calming your breath.

### 2.4. Pulmonary Function Test

The German Jeager Master Screen Body pulmonary function instrument was employed. The patient was instructed to take a sitting position, and the pulmonary function was measured by the instrument after inhaling bronchodilators. Deep inspiratory volume (IC), residual volume (RV), total lung volume (TLC), forced expiratory volume in the first second (FEV1), and forced vital capacity (FVC) were recorded. The percentage of FEV1 in forced expiratory lung capacity (FEV1/FVC %) and residual air volume/total lung volume (RV/TLC) were calculated, and the maximum value was obtained after three repetitions. FEV1/FVC% ≥ 80% was mild; 50% ≤ FEV1/FVC% < 80% was moderate; 30 ≤ FEV1/FVC% < 50% was severe; FEV1/FVC% < 30% was extremely severe.

### 2.5. Data Analysis

SPSS 20.0 was used for data entry and statistical processing. Descriptive statistical analysis was used for the general data of the research objects, and ($\overset{¯}{x}\pm s$) was used for statistical description of the measurement data. The frequency and percentage of counting data were systematically described. *T* test was used to compare the measurement data of normal distribution between groups. Chi-square test was used for comparison between counting data groups, and *P* < 0.05 was considered statistically significant.

## 3. Results

### 3.1. X-Ray Images of Elderly Patients with COPD

Figure 1 showed the image data from a male COPD patient with polymyalgia rheumatica, chronic gastritis, and a history of smoking. Physical examination revealed a blood pressure of 130/79 mmHg, a heart rate of 100 beats/min, a SpO2 of 97%, and a normal heart rate. The abdomen was soft, without tenderness, and no clubs or edema were seen in the extremities. X-ray images showed sparse markings in both lungs, widened anteroposterior diameter of the chest, and emphysema with bullae in both lungs.

Figure 2 showed image data showing a male COPD patient with interstitial lung, hepatic insufficiency, and smoking history. Physical examination revealed blood pressure of 126/79 mmHg, heart rate of 120 beats/min, SpO2 of 94%, and no lymphadenopathy on neck examination. X-ray showed emphysema, decreased lung elasticity, increased retrosternal space, barrel chest, and bullae and interstitial lesions in both lungs.

### 3.2. Comparison of COPD Knowledge between the Two Groups

Before intervention, the average score of COPD knowledge level questionnaire in test group and control group was 20.22 and 21.07 points, respectively, with no statistical significance (*P* > 0.05). After two and four months of intervention, the average score of COPD knowledge questionnaire in the test group was remarkably improved, which was 27.43 points and 30.08 points, respectively, higher than that in the control group (22.79 points and 24.13 points), and the difference was significant (*P* < 0.05, Figure 3).

### 3.3. Comparison of Quality of Life between Two Groups before and after Intervention

Before intervention, the average score of CAT scale in the test group and the control group was 22.31 and 21.45, respectively, with no statistical significance (*P* > 0.05). After two and four months of intervention, the quality of life of patients in the test group was remarkably improved, and the average scores of CAT scale were 18.14 and 14.87, respectively, lower than those in the control group (21.06 and 19.33), with substantial differences (*P* < 0.05, Figure 4).

### 3.4. Comparison of Pulmonary Rehabilitation Training Compliance between Two Groups

Before intervention, there was no substantial difference in compliance between the test group and the control group (*P* > 0.05). Two months after intervention, the number of patients with good compliance in the test group increased significantly. After 4 months of intervention, the number of people with good compliance in the test group increased to 17, and only 1 person had poor compliance. In the control group, only 4 people had good compliance and 24 people had poor compliance; the differences were statistically significant (*P* < 0.05, Figure 5).

### 3.5. Comparison of Self-Efficacy between the Two Groups

Before intervention, the average scores of CSES scale in the test group and the control group were 78.64 and 79.52, respectively, with no statistical significance (*P* > 0.05). After two and four months of intervention, the self-efficacy of patients in the test group was remarkably improved, and the average scores of CSES scale were 103.21 and 107.36, respectively, higher than those in the control group (85.24 and 82.75), with substantial differences (*P* < 0.05, Figure 6).

### 3.6. Comparison of BMI between the Two Groups before and after Intervention

Before intervention, BMI of patients in the test group and control group was 19.23 kg/m^2^ and 19.39 kg/m^2^, respectively, with no statistical significance (*P* > 0.05). After two and four months of intervention, BMI of patients in the test group was also remarkably improved with the improvement of quality of life (20.32 kg/m^2^ and 21.45 kg/m^2^), which were considerably superior to those in the control group (19.76 kg/m^2^ and 20.08 kg/m^2^), and the difference was significant (*P* < 0.05, Figure 7).

### 3.7. Comparison of Exercise Tolerance between the Two Groups

Before intervention, the average length of 6MWD scale in test group and control group was 299.87 m and 300.53 m, respectively, with no statistical significance (*P* > 0.05). After two and four months of intervention, exercise tolerance of patients in the test group was remarkably improved, and the average length of 6MWD scale increased to 328.95 m and 337.62 m, respectively, which were higher than those in the control group (305.24 m and 306.89 m), with substantial differences (*P* < 0.05, Figure 8).

### 3.8. Comparison of Pulmonary Function-Related Indicators between the Two Groups

There were no substantial differences in FEV1, FVC, and FEV1/FVC between the test group and the control group before and after intervention (*P* > 0.05). However, the decrease trend of EV1/FVC in the test group was slower than that in the control group after two and four months of intervention (Figure 9).

## 4. Discussion

The main pathological changes in elderly COPD patients are chronic inflammation of small airways and destruction of lung parenchyma, among which chronic inflammation of small airways is an important factor leading to airflow limitation of small airway remodeling [21–24]. Pulmonary rehabilitation training is one of many exercise exercises for COPD patients and has been proven in clinical trials. Pulmonary rehabilitation training plays a certain role in improving patients' quality of life [25]. Therefore, to further explore the application effect of pulmonary rehabilitation training under 5A nursing mode in elderly COPD patients, a total of 84 patients with chronic obstructive emphysema were included as research objects. The clinical effect of pulmonary rehabilitation training and routine nursing under 5A nursing mode was compared with the corresponding scale. The results showed that before intervention, there was no substantial difference in the average score of COPD knowledge questionnaire between the test group and the control group (*P* > 0.05). After two and four months of intervention, the average score of COPD knowledge questionnaire in the test group was remarkably improved, which was 27.43 points and 30.08 points, respectively, higher than that in the control group (*P* < 0.05). A clear understanding of the related pathological knowledge of COPD in the elderly plays a good role in improving patients' compliance and enthusiasm for coordinated treatment. The pathological knowledge level of COPD in the elderly is affected by the patient's age and education level. Most elderly patients have one-sided knowledge and understanding of diseases, so it is particularly important to strengthen patients' health education in the treatment of diseases [26, 27]. The CSES scale is a commonly used scale to evaluate patients' self-efficacy. The results showed that after two and four months of intervention, the self-efficacy of patients in the test group was remarkably improved, and the average scores of CSES scale were 103.21 and 107.36, respectively, which were considerably superior to those in the control group (*P* < 0.05). Self-efficacy refers to an individual's perception of ability, and the CSES scale is a commonly used self-efficacy scale in clinical practice. The higher the self-efficacy, the higher the patient's recognition and effort of lung health training. Cameron-Tucker et al. (2014) [28] explored the application of chronic disease self-management program (CDSMP) in COPD patients and evaluated exercise self-efficacy, quality of life, self-management behavior, exercise tolerance, etc. The results showed that the chronic disease self-management plan remarkably improved exercise self-efficacy and quality of life of patients, which was in line with the results of this study. Better compliance is an important factor affecting the rehabilitation effect. The lung rehabilitation compliance of two groups of patients before and after intervention was compared. The results showed that two months after intervention, the number of patients with good compliance in the test group increased significantly. After 4 months of intervention, the number of patients with good compliance in the test group increased to 17 and only 1 patient with poor compliance. Lenferink et al. (2017) [29] analyzed the application of self-management interventions in improving the rehabilitation effect of COPD patients, which suggested that better compliance is a key factor in improving the rehabilitation effect of patients, which was in line with the results of this study. Finally, FEV1, FVC, and FEV1/FVC % were compared between the two groups before and after intervention. The results showed that there were no substantial differences in FEV1, FVC, and EV1/FVC% between the test group and the control group before and after intervention (*P* > 0.05). However, EV1/FVC% decreased more in test group than in control group after two and four months of intervention. COPD is a disease with relatively slow progress. The small airway is open during inhalation and closed during exhalation, so there is a difference in the degree of airflow restriction between the inspiratory phase and the expiratory phase, and the small airway forms fixed stenosis with the aggravation of airflow restriction [30]. In this study, although pulmonary function training under 5A nursing mode did not improve airflow limitation significantly, its downward trend was slower than that of conventional nursing.

## 5. Conclusion

In this study, 84 patients with chronic obstructive emphysema were randomly divided into experimental group (pulmonary rehabilitation nursing in 5A mode) and control group (routine nursing), with 42 patients in each group. Through chronic obstructive pulmonary disease knowledge level questionnaire, self-efficacy scale of nurses (CSES), chronic obstructive pulmonary disease assessment test (CAT), 6-minute walking test (6MWD), X-ray image scanning, etc., the results showed that pulmonary rehabilitation training under 5A nursing mode can effectively improve the disease knowledge level, self-efficacy, and compliance of pulmonary rehabilitation training of elderly COPD patients and play an important role in improving the quality of life of patients and alleviating the degree of dyspnea of patients. However, there are some limitations, such as short follow-up time, lack of large sample study, and overall representativeness, so it is necessary to increase the sample size and follow-up time in future studies. Overall, this study provides valid data support for the clinical treatment of elderly patients with COPD.

## Figures and Tables

**Figure 1:** Images of an elderly man (80 years old) with repeated coughing, chest tightness, shortness of breath for 10 years, and aggravation for 1 week.

**Figure 2:** Images of an elderly male (66 years old) who had a 7-day aggravation of imaging images due to repeated coughing and expectoration with chest tightness and shortness of breath for more than 10 years.

**Figure 3:** Comparison of COPD knowledge between the two groups before and after intervention. ^∗^Compared with the test group, *P* < 0.05.

**Figure 4:** Comparison of CAT scores between the two groups before and after intervention. ^∗^Compared with the test group, *P* < 0.05.

**Figure 5:** Comparison of lung rehabilitation compliance between the two groups before and after intervention. (a) Before intervention; (b) 2 months after intervention; (c) 4 months after intervention. ^∗^Compared with the test group, *P* < 0.05.

**Figure 6:** Comparison of CSES scores between the two groups before and after intervention. ^∗^Compared with the test group, *P* < 0.05.

**Figure 7:** Comparison of BMI between the two groups before and after intervention. ^∗^Compared with the test group, *P* < 0.05.

**Figure 8:** Comparison of exercise tolerance between the two groups before and after intervention. ^∗^Compared with the test group, *P* < 0.05.

**Figure 9:** Comparison of mean values of small airway parameters between the two groups before and after intervention. (a) The comparison of FEV1; (b) the comparison of FVC; (c) the comparison of FEV1/FVC.

**Table 1:** Patient assessment items.

Item	Content
COPD knowledge level questionnaire	There are 21 items in the questionnaire. One correct answer is given 2 points, and one wrong answer or no answer is given 0 points. The total score ≥ 28 is grade I. The total score of 14~28 is grade II. An overall score of 14 or less is grade III.
CSES	There are 31 items in the scale, and the higher the score is, the higher the patient's self-efficacy is, including five aspects of emotional management, physical activity management, dyspnea management, safe behavior management, and environment and weather.
CAT	There are 8 items in the questionnaire, and each item is 0 to 5 points. The higher the score, the lower the quality of life. The total score of 0~10 is mild. The total score of 11 to 20 is moderate. The total score of 21 to 30 is severe. An overall score of 31 to 40 is considered extremely severe.

**Table 2:** Guidance programs for different exercise levels.

Sports level	Guidelines
Level 0	Passive training was given priority to, patients were instructed to conduct joint training 1-2 times a day for 15 minutes each time, and patients were assisted to improve ventilation and blood flow ratio by preventing pressure ulcers 1-2 times a day for 15 minutes each time.
Level I	Passive training was given priority to, and patients were instructed to take the semisitting and decubitus position to continue joint activity training, 1~2 times a day, 15 minutes each time
Level II	Based on passive training, the patient's family members were instructed to assist the patient with adaptive training, including regular body position changes, double upper and lower limb activities, and bedside sitting position, 1 to 2 times a day, 15 minutes each time. Patients were instructed to cough effectively for 15 minutes 1-2 times a day.
Level III	Based on auxiliary training and active training, patients were instructed to carry out resistance training, 2-4 times a day, 10 minutes each time. Patient's family was guided to assist the patient with bedside activity training, 1-2 times a day, 10 minutes each time. Patient's family was instructed to assist the patient to stand and continue effective cough training 1-2 times a day for 15 minutes each time.
Level IV	Based on active training, the patient was instructed to sit and stand by the bed and limb resistance training, 1-2 times a day, 15 minutes each time. The patient was also instructed to walk with a walking aid for 15 minutes 2-3 times a day.
Level V	Based on active training, patients were instructed to do resistance training 2-3 times a day for 15 minutes each time. The patient was instructed to walk independently with the aid of a walking aid 2-3 times a day for 15 minutes each time. Meanwhile, the patient was instructed to exercise daily living activities.

## Data Availability

The data used to support the findings of this study are available from the corresponding author upon request.
